The article "RASA1 inhibits the progression of renal cell carcinoma by decreasing the expression of miR-223-3p and promoting the expression of FBXW7" was retracted in 2024. Reasons: plagiarized images; overlap with other authors' work; original data or images not available.

# RASA1 inhibits the progression of renal cell carcinoma by decreasing the expression of miR-223-3p and promoting the expression of *FBXW7*

**DOI:** 10.1042/BSR20194143

**Published:** 2020-07-09

**Authors:** Rui-Li Zhang, Ainiwaer Aimudula, Jiang-Hong Dai, Yong-Xing Bao

**Affiliations:** 1 Postdoctoral Workstation, Changji Branch Hospital of The First Affiliated Hospital of Xinjiang Medical University, Changji, China; 2 Cancer Center, The First Affiliated Hospital of Xinjiang Medical University, Urumqi, China; 3 School of Public Health, Xinjiang Medical University, Urumqi, China

**Keywords:** FBXW7, miR-223-3p, RASA1, Renal cell carcinoma

## Abstract

RAS p21 protein activator 1 (RASA1), also known as p120-RasGAP, is a RasGAP protein that functions as a signaling scaffold protein, regulating pivotal signal cascades. However, its biological mechanism in renal cell carcinoma (RCC) remains unknown. In the present study, *RASA1*, F-box/WD repeat-containing protein 7 (*FBXW7*), and miR-223-3p expression were assessed via quantitative reverse transcription-polymerase chain reaction (qRT-PCR) and Western blot. Then, the targeted correlations of miR-223-3p with *FBXW7* and *RASA1* were verified via a dual-luciferase reporter gene assay. CCK-8, flow cytometry, and Transwell assays were implemented independently to explore the impact of *RASA1* on cell proliferation, apoptosis, migration, and cell cycle progression. Finally, the influence of *RASA1* on tumor formation in RCC was assessed *in vivo* through the analysis of tumor growth in nude mice. Results showed that *FBXW7* and *RASA1* expression were decreased in RCC tissues and cell lines, while miR-223-3p was expressed at a higher level. Additionally, *FBXW7* and *RASA1* inhibited cell proliferation but facilitated the population of RCC cells in the G0/G1 phase. Altogether, *RASA1* may play a key role in the progression of RCC by decreasing miR-223-3p and subsequently increasing *FBXW7* expression.

## Introduction

Renal cell carcinoma (RCC) is a common cancer with approximately 65,000 new cases each year [1]. RCC makes up 2–3% of all adult cancers and ranks eighth among the most common causes of death associated with cancers [2]. Thus, RCC greatly affects quality of life and patient life span while burdening health and economic systems owing to increased risks of metabolic syndrome and cardiovascular and kidney diseases in late stages [3]. Additionally, the incidence and death rate of RCC is increasing worldwide [4]. Thus, studying the molecular basis of RCC is essential for the development of new treatments for RCC patients.

*Ras* small GTPases exert regulatory effects in various signaling cascades as well as in different cellular processes [5,6]. Roughly 30% of human cancers have mutations in *Ras* genes (K-*Ras*, H-*Ras*, and N-*Ras*) making them constantly active in their GTP-bound form [7], giving rise to constitutively active *Ras* signal transduction even without extracellular stimuli. RAS p21 protein activator 1 (RASA1), also known as p120-RasGAP, is a RasGAP protein. In addition to its RasGAP domain, RASA1 has two Src homology 2 (SH2) domains, an SH3 domain, a Pleckstrin homology (PH) domain, and a Calcium-dependent phospholipid-binding (C2) domain. It functions as a signaling scaffold protein regulating pivotal signal cascades [8,9]. RASA1 has also been implicated in many biological processes including actin filament polymerization, blood vessel development, and cell apoptosis and movement [10]. Mice deficient in RASA1 have aberrantly growing blood vessels and exhibit large-scale neuronal apoptosis and embryonic death at E10.5 [11]. In mouse endothelial cells, loss of *RASA1* increases endothelial proliferation and tube formation [10]. Human RASA1 germline mutations are related to an autosomal dominant disorder, capillary malformation-arteriovenous malformation (CM-AVM), featuring malformed atypical capillaries [12]. Despite its physiological functions, the role of *RASA1* in tumor formation, and specifically in RCC, has not yet been elucidated.

The article "RASA1 inhibits the progression of renal cell carcinoma by decreasing the expression of miR-223-3p and promoting the expression of FBXW7" was retracted in 2024. Reasons: plagiarized images; overlap with other authors' work; original data or images not available.

The purpose of the present study was to inquire into the functions of *RASA1* in the occurrence and progression of RCC and to explore its potential mechanisms, in order to provide novel protocols for the diagnosis and therapy of RCC.

## Materials and methods

### Clinical specimens

Renal cancer tissues and corresponding non-cancerous tissues were collected from renal cancer patients who underwent surgical resection at the First Affiliated Hospital of Xinjiang Medical University from 2016 to 2018. All clinical specimens were preserved at -80°C until use. No routine treatments were performed before surgery. All research subjects provided written informed consent in advance, and this project was approved by the Institutional Review Board from the Ethics Committee of the First Affiliated Hospital of Xinjiang Medical University in accordance with the Code of Ethics in the Declaration of Helsinki.

### Cell culture

ACHN, SN12C, 786-0, SKRC-39, A-498 and HTB-46 (RCC cells lines), HK-2 (a normal proximal tubule epithelial cell line), and HEK293T cell lines were purchased from BeNa Culture Collection. The culture medium used contained 10% fetal bovine serum (FBS). Cells were incubated at 37°C in an environment with 5% CO_2_.

### Quantitative real-time PCR (qRT-PCR)

Using manufacturer’s instructions, TRIzol reagent (Invitrogen) was used for total RNA extraction from RCC tissues and cells. Through determination via a NanoDrop 2000 (Thermo Fisher Scientific), 200 ng of RNA from each sample was used for reverse transcription with the ReverTra Ace qPCR RT Kit. THUNDERBIRD SYBR® qPCR Mix (Toyobo) was utilized for the calibration of mRNAs in the three groups through qRT-PCR. Reaction conditions were as follows: 94°C for 2 min, 94°C for 10 s, 56°C for 30 s, 72°C for 1 min, and 72°C for 10 min. The reaction was conducted three times. Finally, with GAPDH and U6 as endogenous controls, mRNA expression levels were normalized to GAPDH expression and quantified via the 2^−ΔΔCt^ method. In addition, miRNA expression was normalized to U6 expression and also quantified via the 2^−ΔΔCt^ method. The qRT-PCR primers used in the present study are listed in Table 1.

The article "RASA1 inhibits the progression of renal cell carcinoma by decreasing the expression of miR-223-3p and promoting the expression of FBXW7" was retracted in 2024. Reasons: plagiarized images; overlap with other authors' work; original data or images not available.

**Table 1:** Primer sequences for qRT-PCR

Gene	Primer sequences	
RASA1	Forward:	5′- ACTTGACAGAACGATAGCAGAAG -3′
	Reverse:	5′- GCCTCCGATCACTCTCTCTTA -3′
FBXW7	Forward:	5′- GTTCCGCTGCCTAATCTTCCT -3′
	Reverse:	5′- CCCTTCAGGGATTCTGTGCC -3′
GAPDH	Forward:	5′-CCATGTTCGTCATGGGTGTGAACCA-3′
	Reverse:	5′-GCCAGTAGAGGCAGGGATGATGTTG-3′
U6	Forward:	5′-CTCGCTTCGGCAGCAGCACATATA-3′
	Reverse:	5′-AAATATGGAACGCTTCACGA-3′
miR-223-3p	Forward:	5′- CAGAAAGCCCAATTCCATCT -3′
	Reverse:	5′- GGGCAAATGGATACCATACC -3′

### Cell transfection and culture

siRNAs targeting *RASA1* or *FBXW7* (F-box and WD repeat domain containing 7), scrambled siRNAs, miR-223-3p inhibitor, miR-223-3p NC inhibitor, miR-223-3p mimic, and miR-223-3p NC mimic were obtained from GenePharma. The pcDNA3.1 plasmid (Thermo Fisher Scientific) was utilized for *RASA1* or *FBXW7* overexpression. Prior to transfection, 786-0 and ACHN cells were trypsinized (0.25%) and inoculated in six-well plates with 1 × 10^5^ cells per well. In the case of 80–90% cell fusion, original medium was replaced with fresh medium lacking serum and antibiotics. Transfection was conducted using Lipofectamine 2000 (Life Technologies Corporation (Gaithersburg, MD, U.S.A.)), followed by cultivation of the transfected cells at 37°C in an environment with 5% CO_2_ for 48 h.

### Dual-luciferase reporter gene assay

Through bioinformatical analysis (miRDB, http://www.mirdb.org/), the targeted association between miR-223-3p and *FBXW7* was predicted. Enzymes were used to digest the *FBXW7* 3′UTR using XbaI. Subsequently, with the use of Lipofectamine 2000 reagent (Invitrogen), HEK293T cells were treated with a pGL3-control luciferase reporter gene vector provided by Promega (Madison, WI, U.S.A.) containing *FBXW7*-wt/*FBXW7*-mut and miR-223-3p mimics/miR-223-3p control. Finally, after 48 h of treatment, a Dual-Glo Luciferase Assay System (Promega) was utilized to examine the luciferase activity in cell lysates following manufacturer's protocols. Each assay was implemented in triplicate at the minimum.

The article "RASA1 inhibits the progression of renal cell carcinoma by decreasing the expression of miR-223-3p and promoting the expression of FBXW7" was retracted in 2024. Reasons: plagiarized images; overlap with other authors' work; original data or images not available.

### CCK-8 assay

In a six-well plate, 10 μl of CCK-8 solution (Dojindo) was added to each fell following cell transfection for 0, 24, 48, and 72 h. Next, the RCC cells underwent 2 h of incubation in a humid chamber with 5% CO_2_ at 37°C. Then, a plate luminometer from Bio-Rad was employed to determine the optical density of the cells at 450 nm. The assay was implemented in triplicate at the minimum.

### Flow cytometry analysis

To analyze the cell cycle, cells were collected from different groups at 24–48 h after transfection, and a cell suspension was obtained by digestion of the cells. The supernatant was removed following centrifugation, the cells were washed in PBS twice to discard any residue, and the cells were immobilized in ethanol (75%) for 4 h at 4°C. Later, the immobilized cells underwent centrifugation and PBS washes, followed by mixing with 40 μg propidium iodide (PI) and 1 ml of a 100 μg RNase staining solution from BD Biosciences, and incubation at room temperature for 15 min. Cell cycle analysis was conducted using a FACSCalibur flow cytometer subsequent to staining, and FACSDiva was adopted for statistical data analysis. In apoptosis assays, transfected cells were obtained from each group and underwent trypsinization (0.25%) 24–48 h later. Following inoculation into 96-well plates (2 × 10^4^ cells per well), 5 μl PI, 200 μl HEPES and 5 μl Annexin V/FITC were added and the mixtures were incubated for 25 min at room temperature. A FACSCalibur FCM from BD Biosciences was used for observing apoptosis. The above three assays were independently implemented to reduce errors, and data were analyzed via FACSDiva software.

### Transwell assay

Matrigel (BD Bioscience) and serum-free DMEM were thoroughly mixed and placed in a Transwell chamber (Corning Incorporated). Cells in serum-free medium at a concentration of 2.5 × 10^4^ cells/ml were placed into the upper chamber (500 μl for each chamber) of 24-well invasion chambers, while culture medium containing 20% FBS was added to the lower chamber. A 4% paraformaldehyde solution was utilized to immobilize the cells, and 0.1% Crystal Violet was used to stain RCC cells after 24–48 h of incubation. Pictures were taken in each chamber, and the cells in 5–10 independent fields were counted. The assay was repeated in triplicate at the minimum.

### Western blot assessment

A BCA Protein Assay Kit from Pierce was utilized to measure the protein concentration of each sample. Following isolation via SDS-polyacrylamide gel electrophoresis (SDS-PAGE) using a 10% gel, the proteins were transferred to a polyvinylidene difluoride (PVDF) membrane provided by Millipore (Billerica) for 120 min. Next, TBST with 5% skim milk was used to seal the membrane, followed by 1 h of incubation with primary antibodies (anti-*FBXW7* and anti-GAPDH) from Abcam and secondary antibody (anti-rabbit IgG H&L) from Abcam at 37°C. An ECL system from Life Technology was used to visualize the antibody signals. Differences in the relative protein levels among samples were detected by GAPDH density as an endogenous control.

The article "RASA1 inhibits the progression of renal cell carcinoma by decreasing the expression of miR-223-3p and promoting the expression of FBXW7" was retracted in 2024. Reasons: plagiarized images; overlap with other authors' work; original data or images not available.

### Nude mouse tumorigenesis experiment

BALB/c nude mice were obtained from Xinjiang Medical University. Animal experiments took place in SPF Animal Laboratory at Xinjiang Medical University. All animal experiments were approved by the Changji Branch Hospital of the First Affiliated Hospital of Xinjiang Medical University. Female athymic BALB/c nude mice were injected with control, NC or RASA1-transfected ACHN cells in the subcutaneous tissue of the right flank. Six nude mice were used per group. Tumor growth was monitored by 2D measurements using electronic calipers starting from the seventh day after tumor transplantation, once every 7 days for a total of 28 days. All surgeries were performed under sodium pentobarbital anesthesia via intraperitoneal injection (40 mg/kg) and all efforts were made to minimize suffering. At 4 weeks post-injection, the mice were anesthetized with 40 mg/kg sodium pentobarbital and then killed by 10% formalin perfusion fixation of central nervous system; death was confirmed by complete cessation of heartbeat and breathing. The tumor tissues were isolated and weighed.

### Statistical analysis

Data from each assay implemented thrice were presented as mean ± standard deviation (SD). The comparison between two different groups with parametric variables was conducted via Student’s *t*-test, while the comparison among multiple groups was performed via one-way ANOVA. GraphPad Prism 6.0 was adopted for statistical processing. *P*<0.05 indicated statistically significant differences.

## Results

### *RASA1* was down-regulated in RCC tissues and cells

*RASA1* mRNA was expressed at lower levels in RCC tissue samples than in adjacent (paracancerous) tissue (Figure 1A). In RCC cell lines, we also found that *RASA1* expression was decreased compared to the HK2 cell line (Figure 1B). Additionally, the RASA1 protein expression, as detected by Western blot, was lower in RCC tumor tissue samples compared with adjacent tissue (Figure 1C).

**Figure 1:** *RASA1* is expressed at lower levels in RCC tissues and cell lines than in control ones (**A**) qRT-PCR manifests that *RASA1* is expressed at lower levels in RCC tissues than in paracancerous tissues. (**B**) Through examination, the expression levels of *RASA1* in six RCC cell lines are found to be reduced relative to those in HK-2 cell line. (**C**) *RASA1* was down-regulated in RCC tissues at protein level. Data are presented as mean ± SD in three independent assays; *P<0.05, ***P<0.001.

The article "RASA1 inhibits the progression of renal cell carcinoma by decreasing the expression of miR-223-3p and promoting the expression of FBXW7" was retracted in 2024. Reasons: plagiarized images; overlap with other authors' work; original data or images not available.

### Effects of *RASA1* on RCC cell apoptosis

The transfection efficiency of the *RASA1* over-expression plasmid was verified in 786-0 cells (Figure 2A). Then, a Western blot was utilized to detect the overexpression of RASA1 and the expression of Caspase 3. Previous studies have reported that Caspase-3 is involved in cell apoptosis. Here, no differences were found in RASA1 and Caspase-3 protein expression between the control cells and NC cells, after *RASA1* transfection. However, the expression of RASA1 and Caspase-3 proteins in cells with *RASA1* overexpression was strikingly increased relative to the NC cells, indicating that RASA1 may regulate Caspase-3 expression and promote cell apoptosis (Figure 2B). To confirm the effect of RASA1 on cell apoptosis, a flow cytometry assay was used to detect apoptosis following *RASA1* overexpression. The results showed that the apoptosis rate increased after *RASA1* overexpression (Figure 2C). These experiments were also performed in ACHN cells and the same results were observed (Figure 2D–F).

**Figure 2:** *RASA1* promotes cell apoptosis (**A**) In 786-0 cells, the expression of *RASA1* is tested by qRT-PCR. (**B**) The expressions of *RASA1* and apoptosis index Caspase-3 are detected by Western blot. (**C**) Flow cytometry is employed to examine the apoptosis rate after overexpression of *RASA1*. (**D**) In ACHN cells, qRT-PCR assay verifies the overexpression efficiency of *RASA1.* (**E**) Western blot is applied to examine the expressions of *RASA1* and Caspase-3. (**F**) Flow cytometry is adopted for examining the apoptosis rate after overexpression of *RASA1*; *P<0.05.

### Influence of *RASA1* on the proliferation, migration, and cell cycle progression of RCC cells

Next, we aimed to verify the influence of *RASA1* on cell proliferation, migration, and cell cycle progression. A CCK-8 assay was conducted which demonstrated that *RASA1* overexpression significantly decreased the viability of 786-0 cells (Figure 3A). Furthermore, a cell colony formation assay disclosed that the rate of colony formation was lower in 786-0 cells with *RASA1* overexpression (Figure 3B). In addition, CCK-8 results showed that overexpression of *RASA1* in 786-0 cells lowered their proliferation ability with a time gradient compared to the NC cells (Figure 3C). A Transwell assay uncovered that *RASA1* overexpression drastically reduced cell migration (Figure 3D). Likewise, *RASA1* overexpression greatly decreased cell proliferation, colony formation, and migration in ACHN cells (Figure 3E–H). Finally, flow cytometry results revealed that *RASA1* overexpression increased the RCC cell proportion in G0/G1 phase in both 786-0 and ACHN cells (Figure 4A,B).

The article "RASA1 inhibits the progression of renal cell carcinoma by decreasing the expression of miR-223-3p and promoting the expression of FBXW7" was retracted in 2024. Reasons: plagiarized images; overlap with other authors' work; original data or images not available.

**Figure 3:** Effects of *RASA1* on the proliferation, migration and cell cycle of RCC cells (**A**) Detection of cell viability after transfection of *RASA1* in 786-0 cells via CCK-8 assay. (**B**) Cell colony formation assay verifies the colony formation rate of 786-0 cells after transfection of *RASA1*. (**C**) Detection of the time gradient effects of *RASA1* on 786-0 cell proliferation via CCK-8 assay. (**D**) Examination of cell migration after transfection of *RASA1* via Transwell assay. (**E**) Examination of cell viability after transfection of *RASA1* in ACHN cells via Transwell assay. (**F**) Cell colony formation assay validates the colony formation rate of ACHN cells after transfection of *RASA1*. (**G**) CCK-8 assay is used to detect the time gradient effects of *RASA1* on the proliferation of ACHN cells. (**H**) Detection of the migration of ACHN cells after transfection of *RASA1* via Transwell assay; *P<0.05.

**Figure 4:** Overexpression of *RASA1* greatly increases RCC cell proportion in G0/G1 phase (**A**) Cell cycle is detected using flow cytometry after overexpression of *RASA1* in 786-0 cells. (**B**) Cell cycle changes are examined by flow cytometry after overexpression of *RASA1* in ACHN cells; *P<0.05.

### RASA1 regulates miR-223-3p

To explore the underlying mechanism of RASA1 in cells, the effect of *RASA1* on the expression of miRNAs closely related to kidney cancer was examined. Here, we assessed miR-132, miR-630, miR-223-3p, miR-508-3p, miR-486, and miR-296-3p [13–19]. *RASA1* overexpression reduced the expression of miR-223-3p (Figure 5A), but had no notable impacts on the expression of other miRNAs tested (Supplementary Figure S1). Next, 786-0 cells were transfected with a miR-223-3p mimic or inhibitor to alter miR-223-3p expression (Figure 5B). A CCK-8 assay showed that miR-223-3p partially reversed the inhibitory effect of RASA1 on cell proliferation (Figure 5C). The effect of miR-223-3p on cell proliferation was also seen in ACHN cells (Figure 5D–F). Further, based on a Transwell assay, miR-223-3p could partially attenuate the inhibition of cell migration caused by *RASA1* overexpression (Figure 5G). The above results indicate that RASA1 might inhibit cell proliferation and migration by regulating miR-223-3p.

The article "RASA1 inhibits the progression of renal cell carcinoma by decreasing the expression of miR-223-3p and promoting the expression of FBXW7" was retracted in 2024. Reasons: plagiarized images; overlap with other authors' work; original data or images not available.

**Figure 5:** *RASA1* functioned by modulating miR-223-3p (**A**) In 786-0 cells, the expression of miR-223-3p is reduced after up-regulating the expression of *RASA1*. (**B**) miR-223-3p mimic and inhibitor transfection efficiency are detected. (**C**) Up-regulation of miR-223-3p can partially reverse the inhibition of *RASA1* on cell proliferation. (**D**) In ACHN cells, the expression of miR-223-3p is reduced after up-regulating the expression of *RASA1.* (**E**) miR-223-3p mimic and inhibitor transfection efficiencies are detected. (**F**) Up-regulation of miR-223-3p can partially reverse the inhibition of *RASA1* on cell proliferation. (**G**) Up-regulation of miR-223-3p in both cell lines partially reverses the inhibitory effect of *RASA1* on cell migration; *P<0.05.

### *FBXW7* is a target of miR-223-3p

Through bioinformatic analysis, *FBXW7* was identified as a potential target gene of miR-223-3p (Figure 6A). There’re some other potential target genes of miR-223-3p, which have high binding scores, but we found they are not dysregulated in RCC tissues. Therefore, *FBXW7* was chosen for the further study. A dual luciferase reporter gene assay confirmed a binding association between FBXW7 and miR-223-3p (Figure 6B,C). Further, we detected the expression level of *FBXW7* mRNA and protein level in RCC tissues. *FBXW7* mRNA and protein were down-regulated in RCC tumor tissues compared with adjacent tissues (Figure 6D,E). Interestingly, the mRNA and protein levels of *FBXW7* were pronouncedly decreased after up-regulation of miR-223-3p expression, but increased when miR-223-3p was down-regulated (Figure 6F–I), confirming that miR-223-3p could modulate the expression of *FBXW7*. In RCC cell lines, the expression of *FBXW7* was generally reduced compared with HK2 cells (Figure 6J). By Pearson correlation analysis, the expression of *FBXW7* was found to be negatively correlated with miR-223-3p expression, but remarkably positively correlated to the expression of *RASA1* in renal cancer tissues, indicating that RASA1 might up-regulate *FBXW7* expression by down-regulating miR-223-3p expression (Figure 6K,L).

**Figure 6:** *FBXW7* is the target gene of miR-223-3p (**A**) *FBXW7* has a potential binding site with miR-223-3p. (**B** and **C**) Dual luciferase reporter gene results in two RCC cell lines. (**D** and **E**) *FBXW7* was down-regulated in RCC tissues at protein level. (**F**) The transfection efficiency of miR-223-3p mimic or inhibitor in 786-0 cells. (**G**) *FBXW7* protein expression is down-regulated after miR-223-3p increment in 786-0 cells, whereas it is elevated after down-regulation of miR-223-3p. (**H**) The transfection efficiency of miR-223-3p mimic or inhibitor in ACHN cells. (**I**) *FBXW7* protein is decreased after up-regulation of miR-223-3p in ACHN cells, while it is increased after down-regulation of miR-223-3p. (**J**) The expression of *FBXW7* is pronouncedly decreased in renal cancer cell lines. (**K**) The expression of *FBXW7* and miR-223-3p are notably negatively correlated in renal cancer tissues. (**L**) *FBXW7* is prominently positively correlated with *RASA1* expression in renal cancer tissues; *P<0.05, **P<0.01.

The article "RASA1 inhibits the progression of renal cell carcinoma by decreasing the expression of miR-223-3p and promoting the expression of FBXW7" was retracted in 2024. Reasons: plagiarized images; overlap with other authors' work; original data or images not available.

### *RASA1* inhibits RCC tumorigenesis *in vivo*

As shown in Figure 7A, overexpression of *RASA1* inhibited tumor growth, while down-regulation of *RASA1* promoted tumor growth *in vivo*, which was confirmed by the detection of tumor volume and weight (Figure 7B,C). Additionally, overexpression of *RASA1* greatly up-regulated the RASA1 protein expression, which was down-regulated with an siRNA targeting *RASA1* in tumor tissues (Figure 7D). Furthermore, Western blot and IHC results revealed that the up-regulation of *RASA1* greatly reduced the expression of Ki67, which was up-regulated when *RASA1* was silenced (Figure 7E,F).

**Figure 7:** *RASA1* inhibited RCC tumorigenesis *in vivo* (**A**) Morphology of tumor xenograft. (**B**) The change in tumor volume was determined every 7 d during the tumor growth. (**C**) Tumor weight of nude mice was significantly increased by the transfection with si-*RASA1* and reduced when *RASA1* overexpressed. (**D**) The protein expression of *RASA1* in each group tumor tissues. (**E**) The protein expression of *Ki-67* in each group tumor tissues. (**F**) The expression of Ki67 in each group tumor tissues was determined by IHC; *P<0.05, **P<0.01, ***P<0.001.

## Discussion

Currently, 14 RasGAPs have been identified in mammals [20], and several of them are epigenetically modified in various cancers [21], including *NF1* [22], *DAB2IP* [23], *RASAL1* [24], and *RASAL2* [25]. Within the RasGAP family, the RASA subfamily is composed of five RasGAPs [21]: RASA1/p120GAP, three GAP1 members (RASA2/GAP1m, RASA3/GAP1IP4BP and RASA4/CAPRI), and RASA5/SynGAP. The RASA group inversely modulates Ras signaling and could therefore curb tumor formation in cancer pathogenesis. The *RASA1* inactive mutation, called a driver mutation, together with the NF1 mutation defines a genetically new subclass of non-small cell lung cancer [26,27]. Allelic deletion of *RASA1* is common in triple-negative breast cancer (BC) with TP53 mutations, and its decrement gives rise to the malignant phenotype of breast cells [28]. However, the role of *RASA1* in RCC remains unclear. The present study disclosed that *RASA1* was down-regulated in RCC tissues and cells. Furthermore, we found that the up-regulation of *RASA1* could inhibit cell proliferation and migration while promoting cell apoptosis. Caspases are cysteine-containing aspartate-specific hydrolases and are the primary executor of cell apoptosis [29]. Caspase-3 is a key protease in mammalian cell apoptosis and is one of the most important proteins in caspase family [30,31]. Here, we demonstrated that RASA1 could promote cell apoptosis by regulating Caspase-3 expression.

The article "RASA1 inhibits the progression of renal cell carcinoma by decreasing the expression of miR-223-3p and promoting the expression of FBXW7" was retracted in 2024. Reasons: plagiarized images; overlap with other authors' work; original data or images not available.

MicroRNAs, non-coding RNAs with 19–22 nucleotides, inversely modulate translation and are implicated in a number of cellular processes. Augmentation of certain miRNAs has been intimately correlated with diverse diseases, including diabetes, obesity, cancers, and cardiovascular diseases [32,33]. Aberrant modulation of miRNAs is an important component in cancers due to both the oncogenic and tumor-suppressive functions of miRNAs [34]. miR-223 is found in the q12 segment of the human X chromosome, whose expression is modulated by transcription factors such as C/EBPa, PU.1, and NFI-A [35]. miR-223 is implicated in modulating functions of the cardiovascular system, human immune system, muscle, and bone [36]. Additionally, miR-223 also functions as a tumor suppressor gene in different tumors. A study by Fabris et al. ascertained that overexpression of miR-223 could inhibit BC relapse through the mediation on the EGF signaling pathway, implying that miR-223 overexpression also has crucial impacts on BC progression [37]. Additionally, it has been ascertained that miR-223-3p promotes cell proliferation and metastasis by down-regulating SLC4A4 in RCC [15]. Here, the expressions of RCC-correlated miRNAs were examined upon *RASA1* overexpression and only miR-223-3p had altered expression. In order to confirm whether *RASA1* regulates miR-223-3p in RCC cells, a rescue experiment was conducted. We found that *RASA1* inhibits cell migration and proliferation but boosts cell apoptosis by inhibiting miR-223-3p expression.

Reports show that miRNAs participate in cell differentiation, apoptosis, and proliferation by targeting downstream mRNAs [38]. It was found in this work that F-box/WD repeat-containing protein 7 (*FBXW7*) is a target gene of miR-223-3p, and is expressed at lower levels in RCC tissues and cell lines. *FBXW7* is pivotal for modulating cell growth and differentiation as well as cell cycle progression in human cells, and its decrement is able to drive cancer cells to proliferate [39,40]. Deletion of *FBXW7* results in poor prognosis in multiple cancers [41,42]. Several recent studies have shown that *FBXW7* is the target of miRNAs and functions in the regulation of cancers. For instance, miR-223 regulates acute lymphoblastic leukemia by suppressing *FBXW7* expression [43]. Additionally, miR-27a promotes lung cancer cell growth by repressing *FBXW7*. These results imply that *FBXW7* acts as a tumor suppressor in human cancers [44]. In the present study, we confirmed an association between miR-223-3p and *FBXW7* by dual-luciferase reporter and found that miR-223-3p regulates the expression of *FBXW7* in RCC cell lines. Moreover, we also found *FBXW7* was overexpressed in RCC tumor tissues and that miR-223-3p and *FBXW7* mRNA expression is negatively correlated, while *RASA1* and *FBXW7* mRNA levels are positively correlated. Hence, miR-223-3p may directly regulate *FBXW7.* Finally, we demonstrated that *RASA1* functions in RCC by regulating miR-223-3p. Taken together, we hypothesize that *RASA1* has a role in the development of RCC by decreasing miR-223-3p expression, thus increasing *FBXW7* expression.

The article "RASA1 inhibits the progression of renal cell carcinoma by decreasing the expression of miR-223-3p and promoting the expression of FBXW7" was retracted in 2024. Reasons: plagiarized images; overlap with other authors' work; original data or images not available.

In conclusion, *RASA1* is lowly expressed in RCC tissues and cell lines and has a role in RCC occurrence and progression by inhibiting the expression of miR-223-3p and enhancing the expression of *FBXW7*. However, the present study has several limitations. First, the sample size was small. Further studies using a large sample size will validate the results shown here. Second, the present study found that *RASA1* can regulate miR-223-3p, but its specific mechanism has not yet been elucidated. Future work will aim to elucidate the mechanism behind RASA1 regulation.

## Supplementary Material

Supplementary Figure S1

## Abbreviations

FBXW7: F-box/WD repeat-containing protein 7
lncRNA: long non-coding RNA
RASA1: RAS p21 protein activator 1
RCC: renal cell carcinoma
